# Image Representational Path of Regional Cultural and Creative Products Based on Genetic Algorithm

This article has been retracted.

**DOI:** 10.1155/2022/5112950

**Published:** 2022-03-15

**Authors:** Baiying Wu, Ruiting Han

**Affiliations:** Department of Fine Arts and Process Design, Yuncheng University, Yuncheng, Shanxi 044000, China

## Abstract

Wenchuang product is the abbreviation of cultural and creative products, which is a modern extension of traditional culture. Its dissemination is conducive to enhancing the popularity, appeal, and influence of Chinese traditional culture. As an important carrier and manifestation of cultural and creative industries, Wenchuang products are the integration of regional cultural industry development and the dominant presentation of regional politics, culture, and economy. As a highly parallel, random, and adaptive search algorithm, genetic algorithm has been widely used in personalized product design, conceptual design, product optimization design, and intelligent design, etc. Based on the genetic algorithm, this paper studies the image representation of regional cultural and creative products. In the field of image representation design of regional cultural and creative products, tree structure coding, real number coding, binary coding, etc. are widely used in this field, and these coding methods all meet the innovative requirements of designers. In the field of image representation design of regional cultural and creative products, genetic coding, as a very important part of applying genetic algorithm, plays a very important role in its research and application.

## 1. Introduction

Cultural and creative industry is an emerging industry with creativity as the core under the background of information economy development in the postindustrial era. Britain, South Korea, the United States, Japan, and other countries have formulated industrial development policies for culture and creativity, which has become a national rejuvenation strategy under economic structure adjustment [1]. Cultural and creative products are the abbreviation of cultural and creative products and the modern extension of traditional culture. Its dissemination is conducive to improving the popularity, appeal, and influence of Chinese traditional culture. As an important carrier and manifestation of cultural and creative industries, cultural and creative products are the integration of the development of regional cultural industries and the explicit presentation of regional politics, culture, and economy [2]. The development path of domestic cultural and creative products is mostly based on practice and lacks the corresponding theoretical basis, which leads to the weak foundation of the development of cultural and creative products, mainly manifested in the formalization of design at the shallow level and the lack of deep understanding of design culture. The design of cultural and creative products should reflect the cultural characteristics of different regions. Regional color is the color preference formed by the long-term historical precipitation of a region due to the influence of religious culture and other factors, which directly reflects the regional characteristics and national culture of the city and helps to improve the identifiability of cultural and creative products and inherit the regional context [3]. The design of cultural and creative products needs to grasp the basic law of innovative design, support the connotation and extension of cultural and creative products with iconology theory, make the image carrier unfamiliar, start from the design origin, create regional cultural characteristics, and show regional cultural confidence. As a model of Chinese traditional color culture, black representing the Earth color after fixation of local river mud and yellow dyed by *Dioscorea* are also important colors in the Chinese traditional five-color system. Its color culture is in one continuous line with Chinese traditional culture, reflecting strong regional characteristics [4, 5].

As a highly parallel, random, and adaptive search algorithm, genetic algorithm has been widely used in personalized product design, conceptual design, product optimization design, and intelligent design. As we all know, growth, reproduction, metabolism, and genetic variation are the basic characteristics of life. The product of evolution is life, which has developed over a long period of evolution to form modern organisms. Through the promotion of materialized entities, the emotional appeal is gradually clear and the regional cultural self-confidence is strengthened, so as to promote the overall development of this region. The premise of building regional cultural self-confidence lies in “cultural identity” [6, 7]. The first aspect is “inheritance,” which is a universal feature of living things; that is, as you sow, you reap. In the process of inheritance, the parent gives the biological information to the offspring, and then the offspring develop and differentiate according to the obtained information, so the offspring always have the same or similar characteristics as the offspring [8]. The execution process of the algorithm is to map the evolutionary individuals to the topological structure, and the genetic operations among individuals are limited in their corresponding neighborhood. According to a certain updating strategy, the global optimal solution can be searched through the interaction among local individuals, which can not only maintain the population diversity, but also have good spatial searching ability, and has been applied in many fields.

Compared with the traditional optimization algorithm, the image performance of genetic algorithm in regional cultural and creative products mainly has the following characteristics [8, 9]. The coding of decision variables is the operation object of genetic algorithm [10]. However, traditional optimization algorithms usually directly determine the actual value of the decision variable itself, but genetic algorithm is a coding form for processing the image representation of regional cultural and creative products. Therefore, we can not only learn from some concepts in biology, such as chromosome and gene, but also imitate the genetic and evolutionary mechanism of organisms in nature. At the same time, it also makes it very convenient for us to apply genetic operators [11, 12]. In the field of image representation design of regional cultural and creative products, genetic coding, as a very important part of the application of genetic algorithm, plays a very important role in its research and application [13, 14]. At present, the coding methods widely used in the field of image representation of regional cultural and creative products include tree structure coding, real number coding, binary coding, etc. These coding methods have well realized the innovative requirements of designers.

## 2. Related Work

Literature [15] suggests that the image representation of regional cultural and creative products not only has cognitive and aesthetic functions, but also can convey the inner feelings of products. Product modeling design mainly refers to the functional modeling of form, and the functionality of modeling includes material function and spiritual function. In [16] through the method of big data analysis, the image representation of regional cultural and creative products usually needs to accumulate a large number of visual symbols and have the basic skills of image visual language and create new modeling elements to express the picture image of the image. Graphic creativity is a process in which new visual symbols are constructed in a certain form and change regularly, so as to endow the image with deeper meaning behind it. Literature [17] shows that regional cultural and creative products transform abstract cultural information into visual image representation and finally convey it to consumers through products. The cultural information here is to take the cultural features and geographical features of a specific place or a specific era as design elements and apply them to products through modern design techniques, so as to finally meet people's spiritual and material needs. Literature [18] proposed that the color adjacency network model was established by extracting and selecting the color of the source image and coloring and adjusting the target color region, and the color scheme was optimized by means of interactive genetic algorithm. In [19] through the method of big data analysis, it is necessary to design the image representation to develop the management system. Literature [20] research shows that the improvement of image representation mainly depends on the powerful logic operation ability and graphics derivation ability of computers, and product modeling design greatly meets the needs of product innovation market and enterprises, making personalized service possible. Literature [21] proposes that image performance is to transmit corresponding information through the visual performance of images. The visual impression of images is better than words. The rational use of image symbols can enable the audience to better understand the ideas contained in images and correctly convey the information behind images. In [22] through the big data analysis method, the image representation of the innovative design method is applied to design the function, modeling, structure, materials, and other aspects of products. Literature [23] research shows that, from the perspective of seeking novelty, the pursuit of unique ideas and ideas for the image performance of regional cultural and creative products is easier to attract people's attention. On the basis of accurate expression of information, more innovative, unique, and different creative designs will make people attracted by graphics and more creative. Personalized graphic information brings people different visual feelings and strengthens people's impression of images. Literature [24] puts forward the image expression of subordinate to graphic art design, and its intuitive expression is the most basic form of expression. Strong visual impact in the design of cultural and creative products is the most basic element to impress consumers. Both have intuitive characteristics.

Based on genetic algorithm, this paper studies the image representation of regional cultural and creative products. There are many ways of design expression, which belong to application category from different categories of design and basic research category from graphic demonstration. Through the discovery, extraction, and creation of graphics, we can find the common features among design categories, and through basic research, starting from the fundamental problems of design, we can go back to the starting point of the problem and explore the cultural significance of the region by using the laws and connotations of design.

## 3. Principle and Algorithm of Genetic Algorithm

To study China's “regional culture,” we should start from the eyes and world outlook of people who identify and define this culture, not from the perspective and understanding of future generations. It simulates the principle of “survival of the fittest” in the biological world and searches the optimal scheme in the maximum range of solution space through genetic algorithm operation. The basic unit of each individual with social relations is its region. The deep cognition and expression of this regional culture carries the connotation of regional cultural self-confidence, which is reflected in the self-confidence of “material space” and “spiritual space” in its environment. Regional cultural self-confidence needs a materialization process, so that social individuals can inherit and carry forward regional excellent culture from explicit understanding. This paper deeply studies the principle of genetic algorithm supporting the image representation design and development process of regional cultural and creative products, gives the overall framework of the image representation system of regional cultural and creative products, divides the functional modules of the system, and gives the implementation process and key steps of the system. The image representation of regional cultural and creative products is one of the core technologies of innovative design. It is a multidisciplinary design technology that pays equal attention to image thinking and logical thinking. By extracting the modeling elements from the typical products of previous dynasties and classifying them according to the product modeling style, this paper constructs the product modeling element information base architecture. Using modern design methods such as genetic algorithm, case-based reasoning, product systematic design, and digital design, an image representation design method of regional cultural and creative products based on genetic algorithm is explored. The image performance of regional cultural and creative products takes the integration of user image as the fundamental starting point, and the key is to collect user image information. Considering that eliminating the product color factor is helpful to the cognitive research of “modeling” image, the color attribute factor is not considered. The research and implementation framework of this method can be divided into the following stages, as shown in Figure 1.

Collection of image representation of regional cultural and creative products: Regional cultural and creative products are mainly collected from the Internet, newspapers, magazines, and other media, while the collection of image performance is obtained by open questionnaire. In the choice of regional cultural and creative products, adjectives covering the “semantic cognitive space” of the products should be selected as much as possible. Through the promotion of materialized entities, the emotional appeal is gradually clear and the regional cultural self-confidence is strengthened, so as to promote the overall development of this region. The premise of building regional cultural self-confidence lies in “cultural identity.” To study China's “regional culture,” we should start from the eyes and world outlook of people who identify and define this culture, not from the perspective and understanding of future generations. The reality is that the cultural and social functions of design have not been stimulated and developed but still remain at the superficial level of formal demand. Excessive interpretation of the decoration and beautification of appearance is used, while it is not comprehensive and systematic analysis of regional noumenon cultural resources from the perspective of local and regional characteristics. The cultural value of graphics is not used, there is no cultural context between different visual subjects, and the information dissemination effect of regional image is scattered. To select regional cultural and creative products, sample cluster analysis test must be carried out first, then the samples are described and analyzed in cognitive space by multidimensional scale method according to the cluster results, and finally the representative product samples are selected by hierarchical cluster analysis based on multidimensional evaluation output data. Establishment of image representation feature unit set: Image representation feature analysis first sets that each product contains several different modeling items, and each image representation item is composed of several image feature units. There is also a tendency in traditional regional culture research; that is, the recognition of psychology and emotion used by people to express the difference between “self” and “the other” in daily life is neglected or regarded as a narrow regional concept or subjective emotional expression, so that the regional division is contrary to tradition and common sense, and it is difficult to gain wide recognition.

Considering the consistency of user evaluation in the population interactive genetic algorithm, based on the quantification of user image preference, the image representation process of interactive regional cultural and creative products is driven by the two aspects of group opinion consensus and satisfaction. The image representation design process is shown in Figure 2.

Genetic algorithm can perform evolutionary calculation not only on the whole product, but also on the parts of the product. For the product whose appearance shape can be divided into independent components, the genetic algorithm with double-layer structure can be used to design the shape of a single component, and then the binary coding genetic algorithm can be used to generate combination schemes for different components. The cultural value of graphics is not used, there is no cultural context between different visual subjects, and the information dissemination effect of regional image is scattered. As the most powerful tool of visual language, the important role of graphics in the expression of regional cultural and creative products lies in the expressiveness of graphics itself. Its more important significance lies in giving play to the cultural responsibility of design, analyzing and presenting regional cultural character by using iconology theory, and establishing a regional image paradigm based on cultural connotation. For the products whose shape modeling cannot be divided into independent components, the main components that have an important impact on the appearance modeling can be selected, and the genetic algorithm with double-layer structure is used for the modeling design of the components. The research framework of image representation optimization design of regional cultural and creative products based on genetic algorithm is shown in Figure 3.

Analysis of the relationship between image semantic set and product modeling feature unit set: The semantic differences between the representative samples selected in the third stage and the representative images selected in the second stage are evaluated again. Through quantitative analysis of the experimental results, the linear quantitative relationship between image semantics and modeling feature units is obtained. This quantitative relationship is embodied in the influence values of different modeling feature units on various image semantics, that is, the contribution values of different modeling feature units to image semantics.

Image semantic set

(1) $$\begin{array}{c} F=\left\{f_{1},f_{2},\ldots ,f_{n}\right\}. \end{array}$$

Contribution value set of regional cultural and creative product feature unit to the *j*-th image semantics

(2) $$\begin{array}{c} A_{j}=\left\{A_{j1},A_{j2},\ldots ,A_{jn}\right\}. \end{array}$$

Item I: image semantic *F*_*j*_ contribution value matrix of regional cultural and creative products

(3) $$\begin{array}{c} A_{ji}=\left[A_{j1}A_{j2},\ldots ,A_{jm}\right]. \end{array}$$

Feature unit set of regional cultural and creative products

(4) $$\begin{array}{c} X=\left\{X_{1},X_{2},\ldots ,X_{n}\right\}. \end{array}$$

Characteristic element matrix corresponding to the *i*-th modeling item

(5) $$\begin{array}{c} X_{i}=\left[X_{i1}X_{i2},\ldots ,X_{im}\right]. \end{array}$$

Then the product's contribution to image semantics FJ is scored

(6) $$\begin{array}{c} y_{i}=\sum_{i=1}^{n}A_{ji}X_{i}^{j}. \end{array}$$

Geometric average of all elements in each row of the matrix

(7) $$\begin{array}{c} {\overset{-}{q}}_{j}=\sqrt[{n}]{\prod_{j=1}^{n}p_{ij}}. \end{array}$$

After ${\overset{-}{q}}_{j}$ is normalized, the weight value *q*_*jo*_ of the total image *e* of the user's expected demand after the image FJ hierarchy analysis is obtained.

Image hierarchy evaluation weight set

(8) $$\begin{array}{c} Q=\left\{q_{1},q_{2},\ldots ,q_{n}\right\}. \end{array}$$

## 4. Image Representation Path of Regional Cultural and Creative Products

### 4.1. Image Representation of Regional Cultural and Creative Products Based on Genetic Algorithm

The reality is that the cultural and social functions of design have not been stimulated and developed but still remain at the superficial level of formal demand. Excessive interpretation of the decoration and beautification of appearance, not comprehensive and systematic analysis of regional noumenon cultural resources from the perspective of local and regional characteristics. It simulates the principle of “survival of the fittest and survival of the fittest” in the biological world and searches the optimal scheme in the maximum range of solution space through genetic algorithm operation. Combination of tradition and modernity: in the public impression, we always think that traditional and regional products are ancient and old and exist in museums for people to watch. To change the public's inherent impression, designers need to inherit the essence of traditional culture in the design of cultural and creative products and integrate products into life with modern design language and modern technology, in order to achieve the perfect integration of tradition and modernity. Regional culture is an individual cultural field under Chinese culture. It develops from the long history of a specific region with local characteristics. It is a culture with local characteristics and a long history. China's design has gone through the process from “technology leading” stage to “market leading” stage. Its background comes from the changes in the economic system of the transition from free planned economy to market economy. With the adjustment of new business economic structure and the rapid promotion of the transformation of old and new kinetic energy, the reality has required it to step into the “innovation leading” stage quickly. Design is regarded not only as the figurative behavior of combining several materials and giving them shape, color, and function for a specific purpose, but also as a process from information analysis to conception and search for the best answer to the problem. The traditional image representation design process of regional cultural and creative products mainly depends on the designer's subjective intuition to search for possible solutions to problems. Due to the limitation of personal ability and time, designers tend to make local optimal solution choices. The image expression of regional cultural and creative products is mainly conveyed by visual function and image thinking, far away from the communication between body and language. This kind of image representation of viewing ahead of regional cultural and creative products has become a new feature of modern urban life. Based on the differences in cognitive angles and methods of genetic algorithms, the concepts of image representation of regional cultural and creative products can be said to vary widely. When designing regional cultural products, we should not only pay attention to the characteristics of regional culture, but also start from the reality of life, so that the design of regional cultural products can be integrated into our daily life, and at the same time, the unique culture can be added into the products, and the spiritual connotation of culture can be displayed on the products through design, thus creating the true value of cultural creative products, not only making the products a cultural carrier, but also serving people's lives, so that more people can be inspired and learn from the design of products while thinking about how to use and explore unique regional cultural resources.

From different perspectives, the perception of images is certainly different. For example, from the perspective of perception, image performance can be divided into realistic image performance and conceptual image performance. However, in terms of generation, image expression can be divided into natural image expression and humanistic image expression. In terms of the correlation between the way of expression and natural objects, image expression can be divided into concrete image expression and abstract image expression. In terms of hierarchy, image representation can be divided into external image representation, internal image representation, material image representation, and so on. Folk art, Ecological Folklore, traditional customs, and other civilized expressions in specific regions are cultural traditions that are still playing a role so far. It is integrated with the environment within a certain geographical range of genetic algorithm, so it is branded with the brand of region. The image performance of regional cultural and creative products is determined according to the characteristics of regional cultural and creative products. For the image performance design of specific products, it is only necessary to distinguish the image performance characteristics of product image performance elements, and it is not necessary to accurately express their image performance characteristics. Therefore, genetic algorithm fuzzy semantic quantization method is generally used to express the image representation feature information of product image representation elements. Using relevant design methods, learn to make full use of regional cultural symbols in modern products, so that modern products reflect regional culture, spread regional characteristic culture, inherit and develop regional culture, enrich the connotation of Chinese culture, increase cultural diversity, and more understand and inherit Chinese culture.

### 4.2. Experimental Results and Analysis

As an important carrier and manifestation of cultural and creative industries, cultural and creative products are the integration of regional cultural industry development and the explicit presentation of regional politics, culture, and economy. The development path of domestic cultural and creative products is mostly practice-oriented, lacking the corresponding theoretical basis, which leads to the weak development foundation of cultural and creative products, mainly manifested in the superficial formalization of design and the lack of deep understanding of design culture. The distribution was compared for three times in the experiment. After 18 generations of interactive genetic evolution operation, a satisfactory progeny population was obtained, and each scheme got a high degree of consensus and evaluation. The changes of the consensus of image representation of regional cultural and creative products and the evaluation level of user groups are shown in Figures 4–6.

The experimental results show that it can be seen from the figure that users' evaluation of color scheme varies greatly in the evolution process of the first 10 generations and tends to be consistent after the 10th generation, which reflects that, with the progress of the algorithm, the cognitive differences of group users are gradually narrowing, and the algorithm presents good convergence. It is often used to simply print some regional cultural symbols and cultural totems on the products. This design method makes the products have a certain degree of recognition, but the expression of culture tends to be superficial. In addition to the expression of color visual image, regional culture, what is more important is the internal value of culture. In the process of creation, image expression is realized and applied to the dissemination of regional culture, so as to materialize regional culture. Graphics is the basic unit of regional culture communication and the “soul” of regional culture. Regional cultural and creative products are derived from the characteristics of graphics, which can make the elements of regional culture expressed explicitly and form an identification system of regional culture from inside to outside and from outside to inside.

The cultural value of graphics is not used, there is no cultural context between different visual subjects, and the information dissemination effect of regional image is scattered. Take the regional brand as an example, the chaos of “getting together” and “being ugly” are frequent, and the regional brand is not scientifically developed under the interdisciplinary system but is randomly pieced together with the well-known elements in the region, and the regional symbols are simply and figuratively copied, and the aesthetic and practical features of the design are replaced by subjective feelings. In order to verify the consistency between the user group's evaluation of the final plan and the calculation results of the model, the distribution was compared for four experiments, and 20 users who had visited the Mausoleum of the First Qin Emperor in Shaanxi Province were selected for evaluation from the aspects of culture and uniqueness. Use triangular fuzzy numbers to collect users' opinions. According to the user's image preference, the consensus degree and the evaluation grades of six color schemes are calculated, as shown in Figures 7–10.

The experimental results show that the consensus degree of user image preference of the five schemes exceeds the threshold 0, and the evaluation level reaches “like” or above. The evaluation grades of scheme 1, scheme 3, and scheme 6 are very like, which is consistent with the optimization scheme calculated from step 1 to step 5, which further verifies the consistency and effectiveness of the actual perception of the user group and the results of the model in this paper. Generally speaking, design is a creative behavior aimed at changing people's lifestyle on the basis of meeting aesthetic needs. The evaluation of its works is carried out by users, the public, and even critics through “image reproduction.” In this process, the author is more like an organizer. He presents the needs in the form of works by using professional and technical means and “recreates” the scheme in combination with the feedback of information. As a design method, image expression pays more attention to the expression of regional ontology consciousness in the context of regional culture, that is, the graphical presentation based on the emotional appeal of “social space,” which is the embodiment of the social value of design. As far as a specific region is concerned, image reproduction is the concretization of regional culture, a dynamic and developing process. It is often used to simply print some regional cultural symbols and cultural totems on the products. This design method makes the products have a certain degree of recognition, but the expression of culture tends to be superficial. While designing regional cultural and creative products, we should not only pay attention to the characteristics of regional culture, but also start from the reality of life, so that the design of regional cultural products can be integrated into our daily life, add unique culture to the products, and show the spiritual connotation of culture on the products through the design, so as to create the real value of cultural and creative products.

## 5. Conclusions

The image expression is mainly based on visual function and image thinking, far away from the communication of body and language. In the process of color matching the introduction of multiuser group participation will help to improve the color matching quality. However, affected by each user's knowledge background, social experience, and personal preferences, the group's preference perception is different. The method of image representation design of regional cultural and creative products based on genetic algorithm proposed in this paper is mainly applicable to the irregular appearance modeling design of simple products, which provides a basis for designers to carry out modeling design. At present, it is mainly used in the field of handicraft design. Regional cultural and creative products based on genetic algorithm belong to the current era. It requires the creator to adhere to the regional culture and traditional culture with emotion and requires the creator to adapt to the new era, new business forms, and new changes with lightning speed, return to the origin, and be specific to the natural space and social space of a specific region; folk art, Ecological Folklore traditional customs, and other civilized expressions are cultural traditions that are still playing a role so far. It is integrated with the environment within a certain geographical range of genetic algorithm, so it is branded with the brand of region.

## Figures and Tables

**Figure 1:** Image representation design method of regional cultural and creative products.

**Figure 2:** Operation flow of image representation scheme of regional cultural and creative products.

**Figure 3:** Image representation optimization design framework of regional cultural and creative products based on genetic algorithm.

**Figure 4:** First change curve of consensus degree and user evaluation level of image performance of regional cultural and creative products.

**Figure 5:** Second change curve of consensus degree and user evaluation level of image performance of regional cultural and creative products.

**Figure 6:** The third change curve of consensus degree and user evaluation level of image performance of regional cultural and creative products.

**Figure 7:** Evaluation level after final scheme consensus degree and consistency decision.

**Figure 8:** Evaluation grade after final scheme consensus and consistency decision.

**Figure 9:** Evaluation level after final scheme consensus degree and consistency decision.

**Figure 10:** Evaluation level after final scheme consensus and consistency decision.

## Data Availability

The datasets used and/or analyzed during the current study are available from the corresponding author on reasonable request.
